The article "Impact of Short-Term Heart Rate Variability in Patients with STEMI Treated by Delayed versus Immediate Stent in Primary Percutaneous Coronary Intervention: A Prospective Cohort Study" was published in 2022. Journal: Comput Math Methods Med.

# Impact of Short-Term Heart Rate Variability in Patients with STEMI Treated by Delayed versus Immediate Stent in Primary Percutaneous Coronary Intervention: A Prospective Cohort Study

**DOI:** 10.1155/2022/2533664

**Published:** 2022-06-20

**Authors:** Shaojie Lin, Xing Yang, Xiaosheng Guo, Jingguang Ye, Xiangming Hu, Haojian Dong, Yingling Zhou

**Affiliations:** ^1^School of Medicine, South China University of Technology, Guangzhou Higher Education Mega Centre, Panyu District, Guangzhou 510006, China; ^2^Guangdong Provincial People's Hospital Zhuhai Hospital, No. 2 Hongyang Road, Jinwan District, Zhuhai 519094, China; ^3^Guangdong Cardiovascular Institute, Guangdong Provincial People's Hospital, Guangdong Academy of Medical Sciences, No. 106 Zhongshan Second Road, Yuexiu District, Guangzhou 510080, China

## Abstract

**Objective:**

Patients with ST-segment elevated myocardial infarction (STEMI) have been treated with the delayed stent strategy to reduce the occurrence of postoperative no-reflow and improve the recovery of postoperative cardiac function. However, the effects of electrocardiac activity and autonomic nerve function after primary percutaneous coronary intervention (pPCI) have been rarely reported. The purpose of this study was to investigate the effects of short-term heart rate variability (HRV) in patients with STEMI treated by immediate stent (IS) and delayed stent (DS) strategy.

**Methods:**

A total of 178 patients with STEMI were divided into 124 cases (69.66%) in the IS group and 54 cases (30.34%) in the DS group from July 2019 to September 2021. The mean heart rate, premature ventricular contraction (PVC), left ventricular ejection fraction (LVEF), left ventricular end-diastolic diameter (LVED), and HRV indexes were compared between the two groups.

**Results:**

In terms of cardiac electrical stability, the number of PVCs, the percentage of PVCs, and the number of paired PVCs in the DS group were lower than those in the IS group. In terms of HRV, high frequency (HF) and standard deviation of all NN (SDNN) intervals were higher in the patients with DS strategy than IS strategy. There were no significant differences in the LVED and LVEF between the two groups.

**Conclusion:**

Compared to the IS strategy, the DS strategy in pPCI in patients with STEMI has advantages in postoperative cardiac electrical stability and short-term cardiac autonomic nerve function, with no difference in postoperative short-term cardiac function.

## 1. Introduction

Acute myocardial infarction (AMI) is characterized by the necrosis of myocardial cells caused by an imbalance in oxygen supply and demand due to severe and sustained ischemia [1]. ST-elevation myocardial infarction (STEMI) is the most common type of AMI, with an increasing incidence and mortality each year [2]. Percutaneous coronary intervention (PCI) is currently the most effective treatment for STEMI [3]. PCI expands the criminal vessel (occlude coronary artery branches that caused myocardial infarction) by expanding balloons and stenting to keep them open, thus ensuring urgent and effective myocardial reperfusion [4]. However, despite the restoration of blood flow to the criminal lesion, stent implantation has the potential to disrupt the intima and induce the formation of distal microthrombi. The delayed stent strategy is proposed as a protective secondary revascularization strategy, which is aimed at allowing the body to restore microvascular function over a relatively long period of time and reduce microcirculation disorders [5]. Previous studies have demonstrated that the use of a delayed stenting (DS) strategy for patients with STEMI with a high thrombus load can reduce the occurrence of postoperative no-reflow and improve the recovery of postoperative cardiac function [6].

The traditional indexes for postmyocardial infarction evaluation mainly include various biomarkers and clinical symptom scores. However, biomarkers are easily affected by age, drugs, and physical or chemical factors, and clinical scores are not objective due to the subjective perceptions of clinicians and patients. Heart rate variability (HRV) can be used to analyze the tens of millisecond differences in the NN interval of each heartbeat due to cardiac sympathetic and vagal interactions [7]. Sympathetic nerve function and vagus nerve function activity change every moment, they antagonize each other, and their balance maintains cardiac autonomic nerve function. And HRV reflects the activity of the cardiac autonomic nerve function [8]. As a reliable predictor of cardiac death, arrhythmias, and sudden cardiac death, HRV is obtained and analyzed in a relatively objective and accurate manner [9–13]. HRV is also a predictor after myocardial infarction, and reductions in SDNN parameters also indicate a poor prognosis [14–17]. Previous research has suggested that primary PCI (pPCI) surgery can recanalize criminal vessels and increase vagal activity while reducing sympathetic activity, thereby improving cardiac autonomic function, leading to an increase in the HRV index after treatment [18]. However, the changes in HRV parameters and cardiac autonomic nervous function after pPCI in patients with STEMI with both the conventional immediate stenting (IS) strategy and DS strategy have not yet been reported. In addition, few studies have compared the occurrence of arrhythmias after the two stent strategies. However, there is controversy regarding the difference in postoperative cardiac function between DS and IS [19]. This study is aimed at investigating the effect of the stenting strategy on HRV, cardiac electrical stability, and cardiac function after pPCI in patients with STEMI. We hope to establish a theoretical basis for the selection of better stent strategies for patients with STEMI through the study of HRV.

## 2. Method

This study is based on a subgroup analysis of a multicenter, open-label, prospective cohort study (prognosis of different stenting strategies in first percutaneous coronary interventions in patients with high thrombus load STEMI, registered at http://www.chictr.org.cn, ChiCTR1800019923). The original study began in January 2018 at three Chinese cardiovascular centers. The three centers are Guangdong Provincial People's Hospital, Guangdong Provincial People's Hospital Zhuhai Hospital, and Jiexi County People's Hospital. The data of this substudy come from the Chest Pain Center of Guangdong Provincial People's Hospital Zhuhai Hospital.

### 2.1. Patients

A total of 178 STEMI patients who underwent pPCI at Guangdong Provincial People's Hospital Zhuhai Hospital from July 2019 to September 2021 were selected and divided into the control group (124 patients in the immediate stent group) and the experimental group (54 patients in the deferred stent group). STEMI patients with the criminal vessel with heavy thrombus burden (thrombus score > 2) and good blood flow (TIMI flow grade 3) after preconditioning (thrombectomy or thrombectomy) received the DS strategy according to the operators (who were blinded to the trial) during pPCI (Figure 1). And other patients would receive IS strategy. All patients received conventional treatment according to the guidelines.

The inclusion criteria were as follows: (1) age ≥ 18 years and definite diagnosis of STEMI, (2) patients undergoing pPCI, (3) signed informed consent, and (4) intraoperative imaging suggesting high thrombus load (thrombus score > 2). The thrombus score was defined as follows: 0 points, no thrombus; 1 point, vague thrombus shadow; 2 points, definite thrombus image, length less than 1/2 of the vessel internal diameter; 3 points, definite thrombus, with a length between 1/2 and 2 times the intravascular diameter; 4 points, determined thrombus length greater than 2 times the intravascular diameter; and 5 points, vascular occlusion, unable to assess thrombus.

The exclusion criteria were as follows: (1) cardiac shock or cardiac arrest, (2) criminal vessel as in-stent occlusion or stenosis or bridge vessel occlusion or stenosis, (3) criminal vessels with entrapment lesions, (4) history of allergy to contrast media, (5) life expectancy of <12 months, and (6) criminal vessel is the left main coronary artery.

### 2.2. STEMI Diagnostic Criteria

The clinical diagnosis of STEMI requires at least two of the following three items: (1) elevation of the ST segment in two consecutive leads of the electrocardiogram (ECG); (2) proportional elevation of cardiac biomarkers after admission, including troponin, creatine kinase (CK), and creatine kinase myocardial band (CK-MB); and (3) typical chest pain symptoms.

### 2.3. Baseline Information

The following data were collected: patient's age, sex, past medical history (including hypertension, diabetes mellitus, myocardial infarction (MI) history, and coronary artery disease (CAD)), family history, personal history (including smoking and drinking history), disease status (including time from patient entry to the hospital door-to-balloon (D to B)), time from symptom onset to balloon (D to B), culprit vessel (including the right coronary (RCA) artery, left anterior descending (LAD) artery, and left circumflex (LCX) artery), number of the diseased vessel and Killip class, and postoperative medications (including use of *β*-blockers). We defined smoking history according to the duration of smoking as the following three conditions: (1) never smoked, (2) quit smoking, and (3) current or quitting less than 1 year. If the patient repeatedly fails to quit smoking, then it will be classified as the third situation.

### 2.4. Physical Examinations and Laboratory Tests

Physical examinations included height, weight, blood pressure, heart rate, respiratory rate, and pulmonary rales. Laboratory tests included troponin I, CK-MB levels, hemoglobin (HGB), blood lipid, preoperative 12-lead/15-lead/18-lead ECG, 24 h ambulatory ECG, and cardiac ultrasound within 72 h postoperation. All patients were tested for HRV within 48 hours after pPCI. The MUSE dynamic ECG monitoring system was used to record at least three lead electrocardiograms for 24 hours, and the results were imported into the MARS analysis system for analysis and statistics (MUSE and MARS are from GE company). We filter invalid signal interference, and if the adjacent NN interval is abnormal or the interference signal exceeds 20%, it will be deleted to ensure that the qualified time of the whole record is not less than 20 hours.

### 2.5. Clinical Evaluation

We compared the heart rate (HR) and HRV index of the two groups after pPCI. According to the Task Force of the European Society of Cardiology and the North American Society of Pacing and Electrophysiology, we assessed both time-domain analysis (TDA) and frequency-domain analysis (FDA) [20]. FDA included very low frequency (VLF), low frequency (LF), and high frequency (HF). TDA is represented by normal to normal (NN) interval, standard deviation of all NN (SDNN) intervals, standard deviation of the averages of NN (SDANN) intervals, average standard deviation of the mean of every 5 min NN (ASDNN) interval, square root of the mean of the sum of the squared differences between adjacent NN (ASDNN), number of pairs of adjacent NN (NN50) intervals differing by >50 ms, and percentage of NN50 (NN50). The HR index includes the mean heart rate, maximum heart rate, minimum heart rate, number of premature ventricular contractions (PVCs), percentage of PVCs (as the percentage of total heartbeats), number of single PVCs, and number of paired PVCs between the IS and DS groups. We also compared cardiac function, including left ventricular ejection fraction (LVEF), left ventricular end-diastolic diameter (LVED), and Killip classification between the two therapies.

### 2.6. Statistics

The SPSS (version 24. 0) statistical software was used for data analysis. The measurement data are expressed as *χ* ± *s* using the *t*-test if they followed a normal distribution or Kolmogorov's method if they did not. And the count data are expressed as rates using *χ*^2^ test. *P* values < 0.05 were considered to indicate a statistically significant difference.

## 3. Results

### 3.1. Baseline

A total of 178 patients with STEMI who underwent PCI at Guangdong Provincial People's Hospital Zhuhai Hospital from July 2019 to September 2021 were selected for enrollment. The baseline characteristics of the included patients were well matched, with a *P* value > 0.05 (Table 1). Their ages ranged from 28 to 83, and 88.76% were male. Among the participants, 124 were treated with the IS strategy, and 54 were treated with the DS strategy during the pPCI (69.66% vs. 30.34%, respectively). There were no significant differences between the two groups in personal history, disease status, and use of postoperative *β*-blockers.

### 3.2. Primary Endpoints

As shown in Table 2, regarding cardiac electrical stability, we found no significant difference in the total number of heartbeats. As for mean heart rate, maximum heart rate, and minimum heart rate, there was no statistical difference between the two groups. However, the number of PVCs (4295.31 ± 13867.98 vs. 1435.89 ± 2506.81, *P* = 0.028), percentage of PVCs (4.96 ± 12.85% vs. 1.46 ± 2.73%, *P* = 0.041), and number of paired PVCs (255.13 ± 909.75 vs. 62.63 ± 85.55, *P* = 0.021) were significantly different between the IS and DS groups.

In terms of the HRV (Table 3), the time-domain parameters in the DS group were longer than those in the IS group, which included SDNN (89.15 ± 26.23 ms vs. 100.67 ± 175.84 ms, *P* = 0.001), SDANN (69.16 ± 25.75 ms vs. 80.74 ± 16.87 ms, *P* = 0.003), and RMMSSD (34.64 ± 17.70 ms vs. 42.43 ± 17.09 ms, *P* = 0.007). Regarding the frequency-domain parameters, VLF, LF, and LF/HF had no difference in the IS group and DS group, while there was a significant difference in HF (10.58 ± 5.31 ms^2^ vs. 14.11 ± 3.87 ms^2^, *P* = 0.011) between the two groups.

### 3.3. Secondary Endpoints

In terms of cardiac function, there was no significant difference in the LVEF (*P* = 0.383) and LVED (*P* = 0.177) between patients with delayed stenting compared with patients with immediate stenting. In addition, the peak CK-MB (*P* = 0.687) and CTnI peak (*P* = 0.450) during hospitalization were not statistically different between the two groups (Table 4).

### 3.4. Subgroup Analysis

During follow-up, we found that some patients with STEMI who received the delayed stent strategy did not actually have stents implanted in the second angiography (*N* = 28, 51.85%). We divided these patients into subgroups according to whether stents were placed on secondary angiography (Table 5). We found that the rate of HF was greater in the no-stent implantation group, while, compared to the stent implantation group, the no-stent implantation group had a longer time in time-domain measures except RMSSD (*P* values < 0.05). The ROC curve of TDA and FDA parameters classified the patients with or without stent implantation in the second angiography. Among all HRV parameters, we found that SDNN had the highest discriminating capacity (AUC 0.8808, 95% CI 0.791-0.970, and *P* < 0.001; Figures 2 and 3). The best cutoff point that identified patients who had stent implantation was an absolute SDNN < 101 ms, with a sensitivity of 67.9% and a specificity of 100%. Similarly, when HRV parameters were included in logistics analysis, SDNN (*P* = 0.032) was also the most relevant to whether stents were used in secondary angiography (Table 6).

## 4. Discussion

### 4.1. Delayed Stent Strategy and Heart Rate Variability

The earliest clinical application of HRV was to assess hypoxia from fetal HRV. In the 1990s, HRV was gradually applied to the prediction and prognosis evaluation of various diseases [20]. And in recent years, HRV parameters have been replaced by faster and more accurate laboratory tests [21, 22]. With the advancement of science and technology, the invention of various new sensors and wearable devices and HRV parameters have become easier to obtain [23, 24]. Moreover, with the increase in the computing power of computing chips, the analysis of HRV has become simple and efficient, and research relating to HRV had also restarted. SDNN and SDANN were strong predictors of cardiac mortality, arrhythmia, and sudden cardiac death after myocardial infarction, independent of other risk factors [25, 26]. A previous cohort clinical trial that included 800 patients showed that the mortality rate was more than five times higher in patients with SDNN < 50 ms than in those with SDNN > 100 ms [27]. A substudy of the ATRAMI trial found that SDNN reduction was a predictor of cardiac mortality [28]. Another retrospective study that enrolled 763 patients found that SDNN was shortened in the MACE group (including death, acute myocardial infarction, and revascularization) compared to the non-MACE group (*P* = 0.01) [12]. Ablonskyte-Dudoniene et al. confirmed that the 5-year risk of cardiac death was nearly ten times higher in patients with low SDANN threshold who were mainly treated with PCI than in patients with high SDANN [13]. Coviello et al. observed lower SDNN and HF values and higher LF values in patients with MACE events than those without [29]. After multivariate analysis, both SDNN and LF before discharge (days 7-10 of hospitalization) were associated with a significantly higher risk of MACE and reinfarction [29]. At a 5-year follow-up, a reduction in SDNN was associated with a 4-fold increase in the risk of nonfatal myocardial infarction. A reduction in SDNN resulted in an increase in the risk of unplanned revascularization by nearly 5-fold. The increase of a series of parameters such as SDNN after pPCI reflected the increase of the activity of the vagus nerve and restoration of the balance of autonomic function. Retroactive research has suggested that in patients with AMI, sympathetic activity is predominant and vagal activity is reduced [15], and this is due to myocardial ischemia stimulating cardiac sympathetic excitatory afferent nerves and causing a more pronounced sympathetic excitation in patients with ischemic cardiomyopathy than in those without. A progressive increase in vagal activity reduces the extent of ventricular arrhythmias. Changes in LF were considered as markers reflecting changes in sympathetic and vagal autonomic nervous system regulation, whereas changes in HF spectral power reflected vagal regulation of cardiac activity. LF/HF is used to assess the balance of autonomic nerve activities and is higher in high-risk patients than in normal patients [30]. In our study, the increase in SDNN and HF in the DS group could be considered beneficial to the balance of autonomic nerve function, which should positively impact the prognosis of patients with STEMI (Table 3). However, large-scale studies, such as DANAMI-3 DEFER, MIMI, and INNOVATION, have all confirmed that the DS strategy cannot reduce postoperative microcirculation disturbance and improve prognosis [19, 31, 32]. The results of our follow-up experiment are in agreement with the abovementioned results. We speculate that with the restoration of blood perfusion, the nerves supplied by the criminal vessels gradually recovered blood supply, the nerve activity gradually returned to normal, and the differences between the two groups disappeared.

### 4.2. Delayed Stent Strategy and Cardiac Electrical Stability

Our study also demonstrated that the number of PVCs, the percentage of PVCs, and the number of paired PVCs were reduced in the DS group compared to the IS group, while the number of single PVCs was not significantly different between the two groups (Table 2). We observed that ventricular arrhythmias were mainly concentrated in the number of PVCs, rather than single PVCs. Multiple PVCs can avoid false-positive results caused by computer misinterpretation and signal interference. In addition to the comparison of the number of PVCs, we also used the percentage of PVCs (the ratio of the number of PVCs to the total number of heartbeats) to reflect the comparison of relative numbers, further excluding the difference in the basal heart rate within-group differences. PVC is an indicator that is easily quantified by computers and less prone to false positives. Compared with other arrhythmia indicators, PVC is chosen as an indicator of cardiac electrical stability, which is more objective and common. Atrial fibrillation, ventricular fibrillation, and other arrhythmias occurred infrequently between the two groups and were not sufficient for analysis and comparison. The main purpose of the index is to further exclude intragroup differences due to differences in basal heart rates. Based on the results of this trial, we hypothesize that the DS strategy is protective against the occurrence of postoperative ventricular arrhythmias. Similar to the IS strategy, the DS strategy ensures sufficient coronary blood flow by effectively opening the criminal vessels, restarting the dormant cardiomyocytes, and avoiding arrhythmias caused by long-term hypoxia and ischemia. At the same time, the DS strategy avoids reinjury of the vascular endothelium during stent placement, thereby reducing the release of inflammatory mediators and the inflammatory response. Therefore, the incidence of premature ventricular contractions was lower in the DS group, which also indicated that the DS strategy could reduce postoperative arrhythmias. Moreover, because of the increase in SDNN and the reduced occurrence of PVCs in the DS group, it suggests that longer time-domain parameters will improve cardiac stability. In another study that enrolled 122 elderly patients with AMI, the group with atrial fibrillation (AF) had a shorter SDNN (110.80 ± 21.38 ms vs. 136.49 ± 27.67 ms, *P* = 0.001) than the group without AF [33]. However, in another clinical study, it involves 138 patients with AMI and postoperative LVEF of less than 35%, SDNN (*P* = 0.018), and HF increased in the nonsudden cardiac arrhythmias (non-SCA) group after AMI compared to those in the SCA group [34]. These findings are consistent with our trial results relating to cardiac electrical stability.

### 4.3. Delayed Stent Strategy and Cardiac Function

No statistical differences were observed regarding the cardiac function indices between the two groups (Table 4). Lønborg et al. showed that the DS strategy did not correlate with the final postoperative infarct size and did not affect microcirculatory flow changes during the period [35]. However, the study by Kelbæk et al. suggested that STEMI patients with DS strategy had a greater increase in LVEF than IS strategy at 18 months postoperatively (60% vs. 57%, *P* = 0.0420) with a trend for the DS group to have a lower percentage of patients with LVEF < 45% (13% vs. 18%, *P* = 0.0506) [19]. Cardiac function parameters were associated with heart rate variability. For example, decreased SDNN values were associated with decreased LVEF. Under normal physiological conditions, the body can regulate the excitation of the vagus nerve and the inhibition of the sympathetic nerve activity through the baroreflex. When the cardiac ejection fraction is sharply reduced, the baroreceptor function is disturbed, which alters the balance between the sympathetic and vagal nerves, resulting in a decrease in SDNN. Some studies have shown that patients with asymptomatic cardiac insufficiency will also experience a decrease in SDNN, and that the SDNN will also decrease with the deterioration of cardiac function [36]. However, the differences in SDNN between the two groups in our study did not lead to differences in LVEF. Because we did not have long-term postoperative monitoring of cardiac function and HRV, it is unclear whether they interact with each other with increasing follow-up time. Therefore, it is presumed that the improvement in cardiac autonomic function with the DS strategy compared to the IS strategy failed to affect the short-term postoperative recovery of cardiac function.

### 4.4. Subgroup Analysis

Some patients in the delayed stent group showed good blood flow conditions at the time of secondary angiography. Our research indicated that the values of HF and TDA parameters in these patients were higher than those of patients with stent implantation during secondary angiography (Table 5). It has been mentioned above that an increase in the value of these parameters indicated a good prognosis. To further test whether these parameters can predict the accuracy of stent implantation in secondary angiography of delayed stents, we plotted AUC for all HRV parameters, with SDNN showing the largest AUC (0.8905) (Figures 2 and 3). We calculated a Youden index of 0.679 and a cutoff value of 101 for SDNN (positive predictive value, 67.9%, and negative predictive value, 100%). The value of SDNN can help the surgeon to make judgments about stent placement during the second angiography.

## 5. Study Limitations

First, this study focused on monitoring autonomic function after pPCI and lacked comparisons for the subsequent intermediate and distant periods. Second, LVEF and LVED were used to assess cardiac function without other imaging support. Third, as a prospective clinical trial, the sample size of the study was insufficient, especially the sample size of the experimental group, and was also limited by single-center and patient compliance. Continuation of the study could be supplemented by including more cases. Forth, the analog signal of the monitoring leads during the patient's postoperative stay in the ICU or CCU was used instead of the traditional 12-lead standard signal; although this reduced the cost during the patient's hospitalization, the accuracy was inferior compared to the traditional standard lead signal. Fifth, we were unable to include intraoperative electrocardiographic data and lacked a time-axis oriented comparison. Sixth, we found that there were very few adverse events during hospitalization in this study, so there was no statistical difference between the two groups. Since the follow-up is still in progress, it is impossible to list all the follow-up data. We hope follow-up data will be compared to HRV in subsequent studies and articles.

## 6. Conclusion

In conclusion, compared to the IS strategy, the DS strategy in pPCI in patients with STEMI has advantages in postoperative cardiac electrical stability and short-term cardiac autonomic nerve function, with no significant difference in postoperative short-term cardiac function.

## Figures and Tables

**Figure 1:** Trail profile. STEMI: ST-segment elevation myocardial infarction; pPCI: primary percutaneous coronary intervention; HRV: heart rate variability.

**Figure 2:** ROC curve of TDA showing the power of classification according to stent implantation or none stent implantation. TDA: time-domain analysis; SDNN: AUC 0.8808, 95% CI 0.791-0.970, and *P* < 0.001.

**Figure 3:** ROC curve of FDA showing the power of classification according to stent implantation or none stent implantation. FDA: frequency-domain analysis.

**Table 1:** Baseline clinical characteristics of participants with the two strategies.

	Participants subjected to IS strategy (*N* = 124)	Participants subjected to DS strategy (*N* = 54)	*P* value
Age (years)	55.94 ± 11.00	53.09 ± 12.94	0.134
Male sex	107 (86.29)	51 (94.44)	0.113
Height (cm)	166.50 ± 6.92	165.56 ± 6.28	0.391
Weight (kg)	68.05 ± 12.83	67.81 ± 13.27	0.856
Hypertension			0.151
Normal or high normal	81 (65.32)	36 (66.67)	
Grade 1	18 (14.51)	7 (12.96)	
Grade 2	6 (4.84)	7 (12.96)	
Grade 3	20 (15.32)	4 (7.41)	
Diabetes mellitus	14 (11.29)	3 (5.56)	0.231
MI history	4 (3.23)	3 (5.56)	0.462
CAD family history	4 (3.23)	4 (7.41)	0.216
Smoking			0.958
Never	28 (22.58)	12 (22.22)	
Quit	12 (9.68)	6 (11.11)	
Current or quitting less than 1 year	84 (67.74)	36 (56.25)	
TG (mmol/L)	1.75 ± 0.83	1.85 ± 0.92	0.168
TC (mmol/L)	5.29 ± 1.18	5.02 ± 1.19	0.491
LDL-C (mmol/L)	3.62 ± 0.84	3.56 ± 0.73	0.655
HDL-C (mmol/L)	1.10 ± 0.36	1.01 ± 0.19	0.073
HGB (g/L)	142.16 ± 18.57	144.93 ± 15.43	0.339
Onset to balloon (min)	336.65 ± 394.41	279.19 ± 188.30	0.190
Door-to-balloon (min)	62.94 ± 28.74	66.80 ± 30.08	0.418
Culprit vessel			
RCA	66 (53.22)	35 (64.81)	0.151
LAD	77 (62.09)	31 (57.40)	0.556
LCX	55 (40.32)	30 (55.56)	0.060
Number of diseased vessels			0.151
1	79 (63.70)	26 (54.55)	
2	22 (17.74)	14 (25.92)	
3	23 (18.54)	14 (25.92)	
Killip class			0.922
I	108 (87.09)	46 (85.18)	
II	8 (6.45)	5 (9.26)	
III	5 (4.32)	2 (3.70)	
IV	3 (2.42)	1 (1.85)	
*β*-Blocker used	82 (66.12)	40 (74.07)	0.294

Data are shown as median (IQR) or *n* (%). IS: immediate stenting; DS: delayed stenting; MI: myocardial infarction; CAD: coronary artery disease; TG: triglycerides; LDL-C: low-density lipoprotein cholesterol; HDL-C: high-density lipoprotein cholesterol; HGB: hemoglobin; RCA: right coronary artery; LAD: left anterior descending artery; LCX: left circumflex artery.

**Table 2:** Heart rate and cardiac electrical stability after pPCI.

	IS group (*N* = 124)	DS group (*N* = 54)	*P* value
Total number of heart beats	107886.75 ± 17344.55	111052.94 ± 29047.22	0.369
Mean heart rate (bpm)	75.38 ± 11.00	77.11 ± 20.19	0.555
Maximum heart rate (bpm)	129.06 ± 28.86	126.04 ± 20.65	0.430
Minimum heart rate (bpm)	44.56 ± 12.23	44.35 ± 14.87	0.921
Number of PVCs	4295.31 ± 13867.98	1435.89 ± 2506.81	0.028
Percentage of PVCs (%)	4.96 ± 12.85	1.46 ± 2.73	0.041
Number of single PVCs	1374.75 ± 3359.44	992.74 ± 1534.69	0.425
Number of paired PVCs	255.13 ± 909.75	62.63 ± 85.55	0.021

IS: immediate stenting; DS: delayed stenting; PVC: premature ventricular contraction; bpm: beats per minute.

**Table 3:** Heart rate variability after pPCI.

	IS group (*N* = 124)	DS group (*N* = 54)	*P* value
Frequency-domain measures			
VLF (ms^2^)	24.71 ± 11.79	24.23 ± 9.23	0.788
LF (ms^2^)	15.36 ± 7.41	16.51 ± 7.69	0.349
HF (ms^2^)	10.58 ± 5.31	14.11 ± 3.87	0.011
5 min total power (ms^2^)	28.94 ± 11.14	28.81 ± 10.34	0.939
LF/HF	1.38 ± 0.58	1.24 ± 0.64	0.163
Time-domain measures			
SDNN (ms)	89.15 ± 26.23	100.67 ± 175.84	0.001
SDANN (ms)	69.16 ± 25.75	80.74 ± 16.87	0.003
ASDNN (ms)	53.32 ± 23.67	59.54 ± 15.55	0.079
RMSSD (ms)	34.64 ± 17.70	42.43 ± 17.09	0.007
pNN50 (%)	8.41 ± 7.35	10.85 ± 9.53	0.066

IS: immediate stenting; DS: delayed stenting; VLF: very low frequency; LF: low frequency; HF: high frequency; NN interval: normal to normal interval; SDNN: standard deviation of all NN intervals; SDANN: standard deviation of the averages of NN intervals; ASDNN: average standard deviation of the mean of every 5 min NN interval; RMSSD: square root of the mean of the sum of the squared differences between adjacent NN; NN50: number of pairs of adjacent NN intervals differing by >50 ms; pNN50: NN50 divided by the total number of all NN intervals.

**Table 4:** Cardiac function after pPCI.

	IS group (*N* = 124)	DS group (*N* = 54)	*P* value
LVEF (%)	52.32 ± 9.42	50.94 ± 10.19	0.383
LVED (cm)	4.85 ± 0.51	4.98 ± 0.78	0.177
Peak of CK-MB (U/L)	291.44 ± 251.12	272.87 ± 342.92	0.687
Peak of cTnI (*μ*g/L)	35217.78 ± 71917.27	27670.65 ± 20553.87	0.450

IS: immediate stenting; DS: delayed stenting; LVEF: left ventricular ejection fraction; LVED: left ventricular end-diastolic diameter; CK-MB: creatine kinase myocardial band.

**Table 5:** Heart rate variability of IS group after second angiography.

	None stent implantation group (*N* = 28)	Stent implantation group (*N* = 26)	*P* value
Frequency-domain measures			
VLF (ms^2^)	23.31 ± 6.25	25.31 ± 11.66	0.416
LF (ms^2^)	16.70 ± 7.94	16.30 ± 7.56	0.850
HF (ms^2^)	15.06 ± 3.67	13.10 ± 3.89	0.063
5 min total power (ms^2^)	27.26 ± 9.28	30.48 ± 11.31	0.872
LF/HF	1.18 ± 0.66	1.31 ± 0.61	0.256
Time-domain measures			
SDNN (ms)	111.39 ± 16.98	89.12 ± 8.75	<0.001
SDANN (ms)	86.46 ± 16.13	74.58 ± 15.67	0.008
ASDNN (ms)	63.82 ± 12.20	54.92 ± 17.58	0.037
RMSSD (ms)	44.50 ± 14.45	40.19 ± 19.57	0.360
pNN50 (%)	14.23 ± 10.76	7.20 ± 6.40	0.006

VLF: very low frequency; LF: low frequency; HF: high frequency; NN interval: normal to normal interval; SDNN: standard deviation of all NN intervals; SDANN: standard deviation of the averages of NN intervals; ASDNN: average standard deviation of the mean of every 5 min NN interval; RMSSD: square root of the mean of the sum of the squared differences between adjacent NN; NN50: number of pairs of adjacent NN intervals differing by >50 ms; pNN50: NN50 divided by the total number of all NN interval.

**Table 6:** Heart rate variability as variables in IS group with logistics.

	*B*	S.E.	Wald	Sig
VLF	0.430	0.251	2.934	0.087
LF	-0.417	0.269	2.399	0.121
HF	-0.785	0.376	4.362	0.037
5 min total power	-0.406	0.244	2.773	0.096
SDNN	-0.535	0.249	4.622	0.032
SDANN	-0.018	0.057	0.098	0.754
ASDNN	-0.088	0.105	0.693	0.405
RMMSD	-0.019	0.102	0.033	0.855
pNN50	-26.372	12.785	4.255	0.039

## Data Availability

The datasets and material used and/or analyzed during the current study are available from the corresponding author on reasonable request.

## Abbreviations

AMI: Acute myocardial infarction
ASDNN: Average standard deviation of the mean of every 5 min NN interval
CAD: Coronary artery disease
CK: Creatine kinase
CK-MB: Creatine kinase myocardial band
DS: Delayed stent
D to B: Door-to-balloon
ECG: Electrocardiogram
HF: High frequency
HGB: Hemoglobin
HR: Heart rate
HRV: Heart rate variability
IS: Immediate stent
LAD: Left anterior descending artery
LCX: Left circumflex artery
LF: Low frequency
LVEF: Left ventricular ejection fraction
LVED: Left ventricular end-diastolic diameter
MI: Myocardial infarction
NN: Normal to normal interval
NN50: Number of pairs of adjacent NN intervals differing by >50 ms
O to B: Onset to balloon
pNN50: Percentage of NN50
pPCI: Primary percutaneous coronary intervention
PVC: Premature ventricular contraction
RCA: Right coronary artery
RMMSD: Square of the root of the mean of the sum of the square differences between adjacent NN
SCA: Sudden cardiac arrhythmias
SDNN: Standard deviation of all NN intervals
SDANN: Standard deviation of the averages of NN intervals
STEMI: ST-segment elevated myocardial infarction
TIMI: Thrombolysis in myocardial infarction
VLF: Very low frequency.
